The article "Biology of Polyomavirus miRNA" was published in 2021. Journal: Front Microbiol.

# Biology of Polyomavirus miRNA

**DOI:** 10.3389/fmicb.2021.662892

**Published:** 2021-04-06

**Authors:** Wei Zou, Michael J. Imperiale

**Affiliations:** Department of Microbiology and Immunology, University of Michigan, Ann Arbor, MI, United States

**Keywords:** polyomavirus, miRNA, persistent infection, virus replication, biomarker

## Abstract

Polyomaviruses are a family of non-enveloped DNA viruses with wide host ranges. Human polyomaviruses typically cause asymptomatic infection and establish persistence but can be reactivated under certain conditions and cause severe diseases. Most well studied polyomaviruses encode a viral miRNA that regulates viral replication and pathogenesis by targeting both viral early genes and host genes. In this review, we summarize the current knowledge of polyomavirus miRNAs involved in virus infection. We review in detail the regulation of polyomavirus miRNA expression, as well as the role polyomavirus miRNAs play in viral pathogenesis by controlling both host and viral gene expression. An overview of the potential application of polyomavirus miRNA as a marker for the progression of polyomaviruses associated diseases and polyomaviruses reactivation is also included.

## General Overview of Polyomavirus Viral miRNA

The *Polyomaviridae* family contains more than 100 members with natural hosts of primarily mammals and birds^1^ (Moens et al., 2017; Ehlers et al., 2019). Polyomavirus genomes have recently also been detected in fish (Van Doorslaer et al., 2018). Each polyomavirus has a very restricted host range and tissue tropism. At present, 14 species have been reported to infect humans, and some clearly cause diseases including polyomavirus-associated nephropathy and hemorrhagic cystitis for human polyomavirus BK (BKPyV), progressive multifocal leukoencephalopathy (PML) for human polyomavirus JC (JCPyV), Merkel cell carcinoma for Merkel cell polyomavirus (MCPyV), and trichodysplasia spinulosa for Trichodysplasia spinulosa-associated polyomavirus (TSPyV). HPyV6 (Human polyomavirus six) has also been linked with chronic pruritic eruptions and Kimura disease, a rare chronic inflammatory disorder that involves subcutaneous tissues (Gardner et al., 1971; Padgett et al., 1971; Haycox et al., 1999; Allander et al., 2007; Gaynor et al., 2007; Feng et al., 2008; Schowalter et al., 2010; van der Meijden et al., 2010; Scuda et al., 2011; Siebrasse et al., 2012; Korup et al., 2013; Lim et al., 2013; Mishra et al., 2014).

One of the most striking observations for human polyomaviruses is the fact that primary infection occurs during childhood, followed normally by lifelong asymptomatic persistence (Wollebo et al., 2015; Imperiale and Jiang, 2016). Periodic virus shedding has been detected in urine of healthy subjects, as has the presence of some viruses on healthy skin, with no clinical symptoms. Serum prevalence studies showed that more than 80% of adults are positive for BKPyV, with variable prevalence for other human polyomaviruses (Stolt et al., 2003; Dalianis et al., 2009; Egli et al., 2009; Kean et al., 2009; Nguyen et al., 2009; Chen et al., 2011; van der Meijden et al., 2011; Nicol et al., 2012; Gossai et al., 2016). Polyomaviruses cause diseases in immunocompromised individuals or transplant recipients who need treatment with immunosuppressive drugs. It remains elusive, however, how the persistent infection enters into a reactivated state with active virus replication upon alterations to the host immune system.

The article "Biology of Polyomavirus miRNA" was published in 2021. Journal: Front Microbiol.

Polyomaviruses contain a circular double stranded DNA genome, approximately 5–6 kb in length, that is divided into an early region, a late region, and a non-coding control region (NCCR), which contains the origin of DNA replication and bi-directional promoters and transcriptional enhancers for early and late region transcription from opposite strands of the genome (Figure 1). The early region encodes large tumor antigen (TAg), small tumor antigen (tAg), and up to three additional tumor antigens through alternative splicing that are important for virus replication and oncogenesis (White et al., 2009; Lagatie et al., 2013; Moens et al., 2017). The late region encodes the capsid proteins VP1, VP2, and VP3 and sometimes a small auxiliary agnoprotein or VP4 that are responsible for virion assembly and nuclear egress (Giorda et al., 2013; Suzuki et al., 2013; Swinscoe, 2019). Based on the NCCR DNA sequence structure, most polyomaviruses including JCPyV and BKPyV include different genotypes which are normally divided into archetype virus and rearranged variants. The archetype virus is thought to be the transmissible, or wild type, form of the virus, which is identified in healthy subjects (in whom the virus establishes a persistent subclinical infection) and in patients with polyomavirus related diseases. Rearranged variants are normally only identified in polyomavirus related disease patients (Doerries, 2006; Gosert et al., 2008).

**FIGURE 1:** Polyomavirus genome map and mechanism of miRNA expression. The dsDNA genome is depicted by the two circles. Inner circle indicates early coding strand; outer circle indicates late coding strand. The locations of the early and late genes are indicated by the thick arrows on the circles. The viral miRNA coding region is indicated as a blue bar: its exact position varies from virus to virus, but it is always complementary to the early region mRNA. NCCR: non-coding control region. Lower left shows miRNA being expressed from the NCCR with processing from an intron derived from tandem transcripts circling more than once. miRNA could also be directly expressed from a primary transcript derived from the NCCR. Lower right shows miRNA expressed from an independent promoter upstream of the miRNA coding region. Forward arrows indicate promoters. LL, leader sequence.

The article "Biology of Polyomavirus miRNA" was published in 2021. Journal: Front Microbiol.

MicroRNAs (miRNAs) are a group of non-coding RNAs with an average of 22 nucleotides that post-transcriptionally regulate gene expression by binding most often to 3′untranslated regions (UTR) of target messenger RNAs (mRNAs) (Ha and Kim, 2014). Typically, miRNAs are encoded in introns of cellular genes, although many viruses also encode miRNAs (Rodriguez et al., 2004; Grundhoff and Sullivan, 2011; Kincaid and Sullivan, 2012). To generate mature miRNAs, a long primary transcript (pri-miRNA) is processed by the Drosha and DGCR8 complex to produce the precursor miRNA (pre-miRNA) (Denli et al., 2004). The pre-miRNAs are exported to the cytoplasm by exportin five and then further processed by the RNase III endonuclease Dicer, resulting in the mature miRNA duplex (Zhang et al., 2004; Okada et al., 2009; Yoda et al., 2010). Both strands derived from the mature miRNA duplex can be loaded into the RNA-induced silencing complex (RISC) consisting of argonaute proteins 1–4 (Meijer et al., 2014; Jo et al., 2015). The target specificity of miRNA is dependent on complementarity between the seed sequence of the miRNA, normally the 5′-most 2–8 nucleotides, and miRNA response elements (MREs) located in the target genes (Lewis et al., 2003; Brennecke et al., 2005; Jo et al., 2015; O’Brien et al., 2018).

A small RNA that we now know to be a miRNA encoded by a polyomavirus was first identified in simian virus 40 (SV40) (Alwine and Khoury, 1980; Sullivan et al., 2005). Since then, all well studied polyomaviruses, including BKPyV, JCPyV, MCPyV, and murine polyomavirus (MuPyV), were shown to encode a miRNA on the late region strand in a location opposite to the early genes (Seo et al., 2008, 2009; Sullivan et al., 2009). Due to the intrinsic property of the double stranded DNA genome of polyomavirus, miRNAs encoded by polyomaviruses are therefore perfectly complementary to the early region and share a universal role in inhibiting early gene expression using an siRNA-like mechanism, although different regions of the early gene are targeted by different polyomavirus miRNAs, correlated with the evolutionary relationship of the viruses (Seo et al., 2008, 2009; Sullivan et al., 2009; Lee et al., 2011; Broekema and Imperiale, 2013; Tian et al., 2014). Both miRNAs (miRNA-3p and miRNA-5p) produced from the pre-miRNA of polyomaviruses function to downregulate the expression of the viral early genes, which is unlike human miRNAs in which one strand of the miRNA duplex is generally degraded (Schwarz et al., 2003). Diverse host genes targeted by polyomavirus miRNAs have also been reported or predicted, hinting at a function of the miRNA in facilitating viral immune evasion (Bauman et al., 2011; Lee et al., 2011; Sung et al., 2014). Polyomavirus miRNAs have also been identified in different biological fluids, including urine, plasma, serum, saliva, and cerebrospinal fluid, from both immunocompromised and healthy individuals (Lagatie et al., 2014; Li et al., 2014; Link et al., 2014; Giovannelli et al., 2015; Pietila et al., 2015; Martelli and Giannecchini, 2017; Martelli et al., 2018a). In this review, we focus on the regulation of polyomavirus miRNA expression, the function of polyomavirus miRNA in viral pathogenesis or oncogenesis, and the potential clinical application of polyomavirus miRNA as a marker for polyomavirus infection or reactivation.

The article "Biology of Polyomavirus miRNA" was published in 2021. Journal: Front Microbiol.

## Regulation of Polyomavirus miRNA Expression

Although most well studied polyomaviruses encode a viral miRNA, how miRNA expression is regulated is poorly understood. Since the NCCR harbors the bi-directional promoter and transcriptional enhancer for both early and late gene transcription, it is not unexpected that studies have shown that the NCCR plays an important role in regulating polyomavirus miRNA expression. Because the polyomavirus miRNA is encoded on the late strand DNA of the viral genome, studies have shown that it was expressed in the late phase of the viral infection (Sullivan et al., 2005, 2009; Seo et al., 2008). However, a study focused on the miRNA function of archetype BKPyV showed that the miRNA is expressed before viral replication begins, indicating an early promoter activity that drives late strand transcription exists to regulate BKPyV miRNA expression. It was proposed, therefore, that the miRNA may restrict viral replication in the archetype virus (Broekema and Imperiale, 2013).

It was also demonstrated, however, that the total amount of miRNA expressed by a rearranged BKPyV is 1,000 times higher than the archetype virus, raising the question of whether the miRNA truly regulates replication (Broekema and Imperiale, 2013). In support of this, mutations in neither the SV40 nor MuPyV miRNA affect viral replication, although in both these cases, rearranged variants were studied (Sullivan et al., 2005, 2009). It was therefore hypothesized that it is the relative amounts of miRNA and early mRNA that govern replication, with the balance favoring miRNA in the archetype virus and mRNA in the rearranged variants. In support of this, flipping the orientation of the NCCR (and, therefore, promoters) in BKPyV confers an archetype phenotype on a rearranged virus, and vice versa (Broekema and Imperiale, 2013). The proposed promoter balance model states that in archetype virus, the NCCR shows weak early promoter activity and strong late promoter activity, which induces high expression levels of viral miRNA. In contrast, a rearranged NCCR exhibits strong early promoter and weak late promoter activity, causing lower levels of miRNA expression (Broekema and Imperiale, 2013).

The article "Biology of Polyomavirus miRNA" was published in 2021. Journal: Front Microbiol.

Although numerous transcription factors (TFs) have been predicted or confirmed to bind to the NCCR of various polyomaviruses to regulate viral early and late gene expression and determine the polyomavirus cell or tissue tropism, few studies have been performed to investigate how viral miRNA expression is regulated by TFs, even though the TFs that could regulate viral late gene expression probably may also control miRNA expression (Yang and You, 2020). Sp1 was among the first TFs identified to bind the NCCR of SV40 and is predicted to bind to the NCCR of all human polyomaviruses (Dynan and Tjian, 1983; Gidoni et al., 1985; Bethge et al., 2015; Ajuh et al., 2018). Of all six Sp1 binding sites in NCCR of SV40, Sp1 mediates early gene transcription by engaging three of them and mediates late gene transcription by engaging the other three sites (Gidoni et al., 1985). Among four Sp1 binding sites in the BKPyV NCCR, mutating the site located proximal to the late gene transcription start site (TSS), SP1-4, activates viral early gene expression, while mutating the Sp1 site proximal to the early gene TSS (SP1-2) inhibits early gene expression in the archetype NCCR (Bethge et al., 2016). Further study showed that an archetype BKPyV harboring a SP1-4 mutation expressed much lower miRNA than the parent archetype BKPyV. Consistent with this finding, decreased miRNA expression was observed in archetype BKPyV but not the SP1-4 mutant after knocking down SP1 expression (Martelli et al., 2018b). The function of TFs that regulate viral late gene expression in regulation of viral miRNA expression warrants further study.

Typically, cellular miRNAs are expressed from introns of protein coding genes (Rodriguez et al., 2004; Kim and Kim, 2007). However, in most primate polyomavirus transcripts no such canonical intron exists from which the miRNA could derive. This question was addressed by a recent study that suggested that during BKPyV late gene transcription, RNA polymerase II circles the genome more than once producing transcripts containing tandem repeats of viral genome sequences. These transcripts could then place the miRNA coding sequence in a genome-sized intron (Zou et al., 2020). Splice junctions that could only be derived from this kind of transcript were identified, and consistent with this observation, the study also showed that a circular DNA template expresses higher levels of viral miRNA than a linear template, which cannot produce tandemly-repeated transcripts (Zou et al., 2020). Polyomavirus viral transcripts circling the genome more than once were also observed during MuPyV and MCPyV infection, due to a weak late strand polyadenylation signal (Adami et al., 1989; Batt and Carmichael, 1995; Theiss et al., 2015). In MuPyV transcripts, a multiple tandem copy of an untranslated 57-bp segment, which was called the leader sequence, was identified at the 5′ end due to the splicing of transcripts circling the genome more than once (Adami et al., 1989). A similar leader-to-leader splice product was also observed in MCPyV-infected PSFK-1 cells (Theiss et al., 2015). All this evidence indicates that polyomaviruses probably use this common strategy to express viral miRNAs (Figure 1).

The article "Biology of Polyomavirus miRNA" was published in 2021. Journal: Front Microbiol.

Strong evidence exists that there are also viral sequences in the genome containing promoter activity that regulate miRNA expression independent of the NCCR (Figure 1). This was confirmed in an MCPyV study that showed an approximately 100 base pair sequence upstream of the miRNA coding region contains a promoter activity that can initiate viral miRNA expression (Theiss et al., 2015). Consistent with this result, ChIP-seq experiments identified an obvious peak of H3K4me3 histone modification, a mark that is strongly enriched at transcriptional start sites, located in this region in addition to the NCCR region. Introduction of synonymous mutations that preserve the TAg coding capacity into this putative promoter abolish the H3K4me3 peak and decrease miRNA expression (Theiss et al., 2015). The authors speculated that the remaining expressed viral miRNA generated from transcripts originated from the NCCR. A recent study on the BKPyV miRNA also suggested that there are sequences both within and outside the NCCR that can regulate miRNA expression (Zou et al., 2020).

Analysis of 643 publicly available JCPyV genome sequences showed that three major miRNA genotypes exist in JCPyV isolates, with some minor variant genotypes. All the mutations located in the miRNA coding region form three single nucleotide polymorphisms (SNPs), with two located in the stem region of the pre-miRNA and one in miRNA-J1-5p. The SNP site located in miRNA-J1-5p does not alter the miRNA seed sequence and no SNPs were identified in miRNA-J1-3p. Interestingly, the SNP located in miRNA-J1-5p changes the TAg amino acid, while the two SNPs located in the stem region are synonymous mutations and cause no amino acid change in TAg (Lagatie et al., 2013). The same miRNA polymorphisms were also observed in JCPyV isolated from blood and urine samples from multiple sclerosis (MS) patients treated with natalizumab, as well as from healthy subjects (Giovannelli et al., 2015; Rocca et al., 2015). Analysis of 298 publicly available BKPyV sequences showed that only one SNP occurs in the miRNA-B1-5p and the loop region, respectively, although multiple variations were identified upstream and downstream the pre-miRNA coding region (Broekema, 2013). Interestingly, no SNP was identified in miRNA-B1-3p corresponding to the miRNA-J1-3p SNP.

The article "Biology of Polyomavirus miRNA" was published in 2021. Journal: Front Microbiol.

Another study focused on miRNA polymorphisms demonstrates that naturally occurring SV40 and JCPyV variants rarely lose miRNA expression. The few variants with insertions or deletions in the miRNA coding region are unable to express viral miRNA due to a defect in the processing of the pri-miRNA by the Drosha complex (Chen et al., 2014). Considering that the BKPyV miRNA-B1-3p and JCPyV miRNA-J1-3p miRNAs are identical, that no SNP has been identified in both miRNA-B1/J1-3p, and that few SNPs have been identified in miRNA-B1/J1-5p (Broekema, 2013; Lagatie et al., 2013), this high degree of sequence conservation strongly suggests that the miRNAs have a very important function during viral infection.

## The Function of Polyomavirus miRNA on Viral Pathogenesis

The functions of polyomavirus miRNAs in viral pathogenesis and latent infection have begun to be elucidated. Due to the intrinsic property of the perfect complementarity to the early gene, the polyomavirus miRNA has a universal role in inhibiting viral T antigen expression in all reported polyomaviruses that encode a miRNA (Seo et al., 2008, 2009; Sullivan et al., 2009; Broekema and Imperiale, 2013; Tian et al., 2014). However, the role of miRNA on viral replication is not consistent for different polyomaviruses. For SV40, a mutant lacking miRNA expression showed similar viral replication as the wild type virus. However, this mutant is more sensitive to cytotoxic T cells lysis and triggers higher cytokine expression than wild type, hinting at the function of miRNA on immune evasion by downregulating TAg expression (Sullivan et al., 2005). Different results were observed in a MuPyV mutant lacking the expression of miRNA. This mutant exhibited the same infection and transformation phenotypes as wild type virus in a mouse model, and in particular the immune response was indistinguishable between the mutant and the wild type virus (Sullivan et al., 2009).

The article "Biology of Polyomavirus miRNA" was published in 2021. Journal: Front Microbiol.

For BKPyV, a miRNA null mutant of a rearranged variant showed no difference in progeny virion production. Of note, however, the same mutation in an archetype virus background results in significantly higher viral replication and progeny production than the wild type virus (Broekema and Imperiale, 2013). This is the first study that showed that a PyV miRNA could regulate virus replication, hinting at a function of the miRNA in regulating virus persistence. Similar results were echoed in a study of SV40 miRNA mutant in a Syrian golden hamster model. Hamsters infected with SV40 mutants unable to express the viral miRNAs in both archetype and rearranged NCCR backgrounds contained higher levels of persistent viral DNA in liver and kidney than animals infected with the wild type viruses (Zhang et al., 2014). However, there was no significant difference in the clearance of the mutants and the wild type viruses by the immune system, arguing that the function of SV40 miRNA in inducing immune evasion is not seen in the hamster host. Interestingly, K661, a naturally occurring miRNA null SV40 with an archetype NCCR structure, showed little difference in virus replication in either immortalized or primary cells compared with a revertant that restored miRNA expression (Chen et al., 2014). This observation is different from that of miRNA function in archetype BKPyV, suggesting that miRNA function is dependent not only on the viral genomic context but also on the cellular and host environment.

A study on MCPyV showed that its miRNA negatively regulates TAg expression like that of other polyomaviruses, and a mutant lacking miRNA expression showed higher viral DNA replication than the wild type virus. More importantly, this mutant lost the ability to establish long term persistence in transfected cells in culture (Theiss et al., 2015). However, MCPyV miRNA is expressed at low levels in 50% of MCPyV-positive MCCs, which is probably due to attenuated NCCR promoter activity during the integration of the MCPyV genome into host chromosome: low expression of MCV-miRM1-5p is not surprising given that TAg expression is required for MCC development, and the miRNA would thus inhibit a required oncoprotein (Lee et al., 2011). Therefore, there may be selective pressure against its expression. The low level of miRNA expression detected in tumor cells is probably derived from a promoter activity of the upstream sequence of the miRNA coding region, which is independent of NCCR. Blocking MCPyV miRNA function has little effect on the tumorigenic activity of T antigens that are expressed from the integrated viral genome (Seo et al., 2009). Interestingly, a recent study showed that a major high abundant circular RNA was encoded in the early region opposite to the MCPyV miRNA coding region. The circular RNA can be targeted by miRNA and played a sponge role to regulate viral early gene expression (Abere et al., 2020). Together, this argues for a role of the miRNA of MCPyV in the development of MCC.

The article "Biology of Polyomavirus miRNA" was published in 2021. Journal: Front Microbiol.

In contrast to the low expression level of MCPyV miRNA in MCC, the miRNA expressed by a racoon polyomavirus (RacPyV) is highly abundant in RacPyV-associated neuroglial brain tumors (Dela Cruz et al., 2013; Chen et al., 2015). Although this miRNA presumably inhibits early gene expression, high levels of TAg mRNA were detected in the primary tumor tissues (Brostoff et al., 2014). This work was the first description of a polyomavirus miRNA that is abundantly expressed in tumors, raising the question of how the miRNA expression was regulated and the relationship between the viral miRNA and the tumorigenesis. One possible reason is that the RacPyV genome exists as an episome in the tumors (Dela Cruz et al., 2013), which is different from MCPyV in which the genome is inserted into the host genome (Feng et al., 2008), and therefore presumably maintains the full function of the NCCR promoter activity. As such, promoter balance may still favor oncogene expression, with the RacPyV working as a rearranged variant that expresses high level of both TAg and miRNA.

Studies have also shown that Skp-F-box-cullin (SCF) E3 ubiquitin ligase family members including Fbw7, βTrCP, and Skp2 induce the degradation of TAg protein and maintain MCPyV persistent infection (Kwun et al., 2017). However, tAg of MCPyV inhibits Fbw7 E3 ligase and promotes stabilization of the TAg protein (Kwun et al., 2013). Therefore, it is likely that polyomavirus persistent infection is accomplished by complicated interactions between viral miRNAs, viral tumor antigens, and host factors.

Identification of the host targets of polyomavirus miRNAs is a useful strategy to understand the function of the viral miRNAs in polyomavirus pathogenesis or oncogenesis. However, at present, only a few miRNA host targets have been identified or predicted. The JCPyV and BKPyV 3p-miRNAs, which are identical, have been reported to facilitate viral immune evasion by specifically downregulating the expression of ULBP3, a stress-induced ligand that is recognized by the killer receptor NKG2D, to avoid recognition by NK cells or CD8+ T cells (Bauman et al., 2011). Of note, evidence exists that viral miRNAs derived from EBV, KSHV, and HCMV target another NKG2D ligand, MICB, to escape NKG2D-mediated killing by NK cells (Stern-Ginossar et al., 2007; Nachmani et al., 2009). Studies on MuPyV showed that the viral miRNA targets Smad2, a pro-apoptotic factor, to suppress apoptosis and facilitate virus replication (Sung et al., 2014). Another study showed that a mutant of MuPyV lacking miRNA expression sheds significantly lower levels of viral DNA than the wild type virus in mice, and the defect is largely recovered during infection of immunodeficient mice (Burke et al., 2018). This result indicates that the MuPyV miRNA promotes viral shedding during infection through an unknown mechanism, perhaps to evade host adaptive immune response and/or to promote viruria (Burke et al., 2018). Several host genes were predicted to be MCPyV miRNA targets, which could contribute to the MCC phenotype (Lee et al., 2011). However, the MCPyV miRNA was only detected in half of MCC tumors, with very low expression levels, suggesting that the viral miRNAs might not function in development of MCC (Lee et al., 2011).

The article "Biology of Polyomavirus miRNA" was published in 2021. Journal: Front Microbiol.

As discussed above, the main difference between archetype viruses and rearranged variants is the structure of the NCCR (Broekema et al., 2010). NCCR rearrangements are part of an adaptation strategy of polyomaviruses necessary for efficient replication in diverse cell types (Moens and Van Ghelue, 2005). For example, JCPyV isolates with archetype NCCRs are shed in the urine of healthy and diseased individuals, whereas isolates with a rearranged NCCR are generally recovered from the brain and cerebrospinal fluid of patients with PML (Takahashi et al., 2020). The emergence of BKPyV with rearranged NCCRs is mostly linked to BKPyV-associated nephropathy disease in kidney transplant recipients (Gosert et al., 2008). The rearranged NCCR reflects the ability of polyomavirus to adapt to new cellular environments with broader host cell tropism and permissivity, and higher viral gene expression and replication than that of archetype virus. However, polyomavirus miRNAs exert less of an effect on inhibiting rearranged virus replication as noted above, as the accumulation of TAg from rearranged polyomaviruses offsets the inhibitory effect of the viral miRNA. This is consistent with the observation that miRNA-null rearranged BKPyV and MuPyV show no difference in viral replication compared with the wild type virus, and the RacPyV tumors display both high TAg and miRNA (Sullivan et al., 2009; Broekema and Imperiale, 2013; Brostoff et al., 2014). Polyomavirus miRNA, like other miRNAs in general, probably works as a fine tuner which is likely to be of significance to the establishment, maintenance, and/or reactivation of persistent infections in susceptible hosts by viruses that commonly establish chronic infections.

## Potential Application of Polyomavirus miRNA as a Biomarker for Polyomavirus Infection or Reactivation

In recent years, increasing evidence has suggested that polyomaviruses take advantage of exosomes (or extracellular vesicles) for viral transmission and spread, including JCPyV and BKPyV (Morris-Love et al., 2019; Handala et al., 2020). The viruses packaged in exosomes maintain high infectivity, perhaps more infectious than purified viruses, and the infection is not affected by removing the cellular receptor. However, exosome-packaged JCPyV and BKPyV displayed different sensitivity to antiviral sera. JCPyV packaged in exosomes is not inhibited by JCPyV-specific antisera compared to purified viruses, while BKPyV in exosomes is efficiently inhibited by neutralizing antibody. The data indicate that the neutralizing antibody could neutralize both the BKPyV packaged in exosomes and purified viruses after a 4 h inoculation, suggesting the neutralization happens after viral internalization and endocytosis (Morris-Love et al., 2019; Handala et al., 2020). Polyomavirus miRNA has also been detected at variable levels in exosomes derived from virus infected cells and clinical fluids including urine, plasma, serum, cerebrospinal fluid (CSF) and saliva originating from immunosuppressed patients, and healthy subjects (Giovannelli et al., 2015; Rocca et al., 2015; Kim et al., 2017; Martelli and Giannecchini, 2017; Martelli et al., 2018b). Studies have shown that laboratory and clinical rearranged BKPyV strains show higher replication rates but significantly lower miRNA levels than archetype virus, both intracellularly and in exosomes (Martelli et al., 2018b). Among urine-derived exosome samples from patients shedding BKPyV, lower levels of miRNA-5p were detected in the context of rearranged NCCR variants than in the setting of an archetype NCCR (Martelli et al., 2018b). It was also reported that BKPyV miRNA was highly abundant in exosomes derived from urine in patients with BKPyV nephropathy (Kim et al., 2017).

The article "Biology of Polyomavirus miRNA" was published in 2021. Journal: Front Microbiol.

For JCPyV, detection of viral DNA in plasma (viremia) is rare and has been shown not to be useful for predicting PML (Berger et al., 2013; Major et al., 2013a,b; Subramanyam et al., 2013). As the risk of developing PML among MS patients increases upon prolonged treatment with the immunosuppressive drug, natalizumab, current guidelines recommend discontinuation of natalizumab use in JCPyV seropositive patients (Sormani and De Stefano, 2014; Kornek, 2015). However, due to the high prevalence of JCPyV antibodies in the general population, seropositivity is not sufficient to assess risk or to justify whether natalizumab should be used since not all seropositive MS patients have the same risk of developing PML (Delbue et al., 2015). Therefore, investigations have been conducted to examine the presence of JCPyV miRNAs expression in subjects with low and high risk for PML (Rocca et al., 2015; Takahashi et al., 2020). In immunosuppressed patients, JCPyV miRNA was detected in 6% of plasma sample-derived exosomes in the absence of PML, with a much higher positivity in 43% of serum samples and 60% of CSF-derived exosomes from PML patients (Rocca et al., 2015). High levels of JCPyV miRNA were also detected in PML tissue samples (Takahashi et al., 2020). However, the JCPyV miRNA was also detected with high prevalence in healthy individuals, including in both serum-positive and negative samples (Lagatie et al., 2014). Therefore, the application of JCPyV miRNA as a diagnostic marker to assess the progression of JCPyV-associated diseases or the development of PML needs further comprehensive studies.

Increasing evidence has suggested a connection between human polyomaviruses and infections of the respiratory tract and oral cavity. Many of human polyomaviruses including JCPyV, BKPyV, MCPyV, HPyV6, KIPyV, and WUPyV have been isolated from or detected in tonsils, salivary glands, and/or respiratory secretions (Robaina et al., 2013; Link et al., 2014; Martelli and Giannecchini, 2017; Martelli et al., 2018a). The expression of BKPyV, JCPyV, and MCPyV miRNAs and viral DNA was detected in saliva and plasma samples of 100 HIV-infected patients and 50 healthy subjects. Overall, the polyomavirus miRNA in saliva samples showed a higher prevalence (65%) than that in both paired plasma samples (41%) and also as compared to polyomavirus DNA (24%) (Martelli et al., 2018a). Although no prevalence difference of polyomavirus DNA or miRNA was detected between HIV positive patients and healthy controls, in miRNA saliva-positive samples, all polyomaviruses detected showed lower miRNA levels in healthy subjects compared with that in HIV patients. Likewise, in viral genome saliva-positive samples, all polyomaviruses tested showed lower viral titers in healthy subjects compared with that in HIV patients. Combined with the results that miRNA showed a much higher prevalence than viral DNA and the miRNA prevalence in saliva is much higher than that of plasma, this makes saliva an ideal sample and miRNA a better diagnostic marker for testing polyomavirus infection (Martelli et al., 2018a).

Since JCPyV and BKPyV miRNA have been detected in the plasma, urine, and CSF of immunocompromised patients and healthy subjects, with similar detection rates in PyV-seropositive and PyV-seronegative subjects, all these data suggest polyomavirus miRNA may be a surrogate marker for polyomavirus associated disease (Robaina et al., 2013; Link et al., 2014; Pietila et al., 2015; Kim et al., 2017; Martelli and Giannecchini, 2017; Martelli et al., 2018a). However, miRNA levels vary significantly in seropositive or seronegative subjects; in viral DNA positive or negative subjects; and in polyomavirus-associated disease patients, immunocompromised patients, and healthy subjects. Since polyomavirus DNA positive subjects also harbor archetype and/or rearranged variants, it is difficult to conclude whether there is a function of the miRNA during polyomavirus reactivation and the progression of polyomavirus associated diseases. Although most experiments quantify polyomavirus miRNA through stem-loop qPCR, different criteria (Ct values) have been used to define positivity. Different methods for treatment of the samples and different reaction systems also increase the amount of variation. Since there is a high degree of homology of the miRNA sequences between some polyomaviruses, cross-reaction of different viral miRNAs may also affect the perceived prevalence (Lagatie et al., 2013). Archetype and rearranged polyomaviruses showed very large differences in viral miRNA expression and its relationship with polyomavirus associated diseases, but few studies investigated how the miRNA levels vary with respect to the genotype of the NCCR. Whether and how polyomavirus miRNAs may serve as a marker for polyomavirus diseases or polyomavirus reactivation requires further investigation.

The article "Biology of Polyomavirus miRNA" was published in 2021. Journal: Front Microbiol.

## Conclusion

miRNAs post-transcriptionally regulate gene expression and play an important role in a variety of biological processes including development, cell growth and differentiation, survival, regulation of apoptosis, oncogenesis, and viral infection (Kincaid and Sullivan, 2012; Fu et al., 2013; Hayes et al., 2014; Tufekci et al., 2014). Most polyomaviruses establish lifelong persistence, which requires host immune evasion (Lau et al., 2015; Imperiale and Jiang, 2016). Since they are caused by opportunistic pathogens, most polyomavirus-associated diseases result from dysregulated control of persistent infection, mostly due to immune system suppression leading to reactivation of polyomaviruses. With the implementation of more potent immunosuppressive drugs in the last three decades, polyomavirus has posed an increasing threat to human health (Helle et al., 2017). Of no doubt, increasing evidence demonstrates the important roles of polyomavirus miRNA in polyomavirus persistence and immune evasion. Since rearranged polyomavirus variants are believed to be the causal agents of many polyomavirus related diseases, and viral miRNAs display different functions in the replication of archetype and rearranged variants, continued deciphering of the biological activities of polyomavirus miRNAs will shed light on understanding the pathogenesis of these viruses. Since there are no FDA-approved drugs for treating polyomavirus-associated diseases, investigating the role of polyomavirus miRNAs in viral pathogenesis has the potential to identify novel therapeutic targets for treatment of these patients.

The article "Biology of Polyomavirus miRNA" was published in 2021. Journal: Front Microbiol.

## Author Contributions

WZ wrote the first draft and edited subsequent the versions. MI edited the versions. Both authors contributed to the article and approved the submitted version.

## Conflict of Interest

The authors declare that the research was conducted in the absence of any commercial or financial relationships that could be construed as a potential conflict of interest.

## Footnotes

1 ictvonline.org
